# Schizandrin A exerts anti-tumor effects on A375 cells by down-regulating H19

**DOI:** 10.1590/1414-431X20198385

**Published:** 2019-10-10

**Authors:** Yiming Bi, Yan Fu, Shuyan Wang, Xingxiu Chen, Xiaoping Cai

**Affiliations:** 1 Department of Oncology, Binzhou People's Hospital, Binzhou, China; 2 Department of Dermatology, Binzhou People's Hospital, Binzhou, China

**Keywords:** Malignant melanoma, Schizandrin A, H19, PI3K/AKT

## Abstract

Malignant melanoma (MM) is one of the malignant tumors with highly metastatic and aggressive biological actions. Schizandrin A (SchA) is a bioactive lignin compound with strong anti-oxidant and anti-aging properties, which is stable at room temperature and is often stored in a cool dry place. Hence, we investigated the effects of SchA on MM cell line A375 and its underlying mechanism. A375 cells were used to construct an *in vitro* MM cell model. Cell viability, proliferation, apoptosis, and migration were detected by Cell Counting Kit-8, BrdU assay, flow cytometry, and transwell two-chamber assay, respectively. The cell cycle-related protein cyclin D1 and cell apoptotic proteins (Bcl-2, Bax, cleaved-caspase-3, and cleaved-caspase-9) were analyzed by western blot. Alteration of H19 expression was achieved by transfecting with pEX-H19. PI3K/AKT pathway was measured by detecting phosphorylation of PI3K and AKT. SchA significantly decreased cell viability in a dose-dependent manner. Furthermore, SchA inhibited cell proliferation and cyclin D1 expression. SchA increased cell apoptosis along with the up-regulation of pro-apoptotic proteins (cleaved-caspase-3, cleaved-caspase-9, and Bax) and the down-regulation of anti-apoptotic protein (Bcl-2). Besides, SchA decreased migration and down-regulated matrix metalloproteinases (MMP)-2 and MMP-9. SchA down-regulated lncRNA H19. Overexpression of H19 blockaded the inhibitory effects of SchA on A375 cells. SchA decreased the phosphorylation of PI3K and AKT while H19 overexpression promoted the phosphorylation of PI3K and AKT. SchA inhibited A375 cell growth, migration, and the PI3K/AKT pathway through down-regulating H19.

## Introduction

Malignant melanoma (MM) is one of the malignant tumors with highly metastatic and aggressive biological actions. Besides, MM accounted for 60–80% of skin-cancer related deaths (1). Recent studies have indicated that MM is not a single entity but a set of various kinds of neoplasms with different causes, biological behaviors, and outcomes (2). Unfortunately, despite the development of technology and medicine, the survival rate for advanced MM has not improved significantly in the past eight years (3). Therefore, new medicines or therapies are urgently needed to treat MM. In recent years, more attention has been given to traditional Chinese medicine for novel potential treatment.

Schizandrin A (SchA), extracted from *Fructus schisandra*, has been proven to play effective functions in various diseases due to its biological properties (4). For example, SchA alleviated lipopolysaccharide-induced inflammatory injury in human keratinocyte HaCat cells (5). SchA increased chemosensitivity to 5-fluorouracil by upregulation of miR-195 in colon cancer cells (6). Importantly, previous studies have reported that SchA possesses anti-tumor activities (7). Hence, we hypothesized that SchA might play a vital role in MM.

In recent years, long non-coding RNAs (lncRNAs) have received considerable attention due to their important functions in regulating gene expression in multiple approaches, such as chromosome remodeling, transcription, and post-transcriptional processing (8). Increasing evidence has proven that lncRNAs are closely associated with tumor development or progression (9). For example, lncRNA plasmacytoma variant translocation 1 (PVT1) participates in prostate cancer cell development and growth (10). LncRNA maternally expressed gene (MEG) 3 alleviates gastric cancer cell proliferation and metastasis (10). Among all the identified lncRNAs, lncRNA H19 was characterized as an oncogenic gene in diverse cancers, and the potentiated expression of H19 is closely related to tumor genesis and development (11). Importantly, lncRNA H19 was reported to promote glucose metabolism and cell growth in MM through regulating miR-106a-5p/E2F3 axis (12). Furthermore, the elevated expression of lncRNA H19 predicted poor outcomes for MM via regulating cell growth, invasion, and migration (13). Therefore, we inferred that SchA might play its roles in MM cell lines through regulating lncRNA H19.

In our study, we used A375 cells to construct a MM model *in vitro* and investigated the effects of SchA on A375 cells and its underlying mechanisms.

## Material and Methods

### Cell culture and treatment

The MM cell line A375 (ATCC^®^ CRL-1619™) was purchased from American Type Culture Collection (ATCC, USA). The culture medium for A375 cells was Dulbecco's modified Eagle's medium (DMEM, ATCC, Cat. No. 30-2002) supplemented with 10% fetal bovine serum (FBS, Gibco, USA). The cells were maintained in the environment with 5% CO_2_ and 37°C.

SchA (≥98.0% (HPLC), Figure 1) was obtained from Sigma-Aldrich (USA). SchA was diluted in dimethylsulfoxide (DMSO) to 0–50 μM. The cells were treated with SchA for 24 h.

**Figure 1.** Molecular formula of schizandrin A.

### Cell viability assay

Cell Counting Kit-8 (CCK-8, Yeasen, China) was used for examining cell viability. Treated A375 cells were seeded in a 96-well plate at the density of 2×10^5^ cells/well, under proper conditions (37°C and 5% CO_2_). Then, 10 μL CCK-8 solution was added and cells were incubated for 1 h. After incubation, absorption was read at 450 nm using a Microplate Reader (Bio-Rad, USA).

### Proliferation assay

Bromodeoxyuridine (BrdU, Sigma-Aldrich) was used for cell proliferation assay. In brief, A375 cells treated with SchA or co-treated with SchA and transfected with pEX-H19 were plated in a 96-well plate. Then, BrdU (1 mg/mL) was added to the cultured cells. Cells were then incubated for 3 h and proliferated cells were labeled. Finally, cells incorporated with BrdU were quantified using a BrdU cell proliferation assay kit (Roche Diagnostics, USA).

### Cell apoptosis assay

Propidium iodide (PI) and fluorescein isothiocyanate (FITC)-conjugated annexin V staining (Yeasen, China) were used for cell apoptosis assay. In brief, cells at the density of 100,000 cells/well were seeded in a 6-well plate. Treated cells were washed twice with precooled phosphate buffer saline (PBS) and resuspended in binding buffer. Then, 5 μL annexin V-FITC was added and mixed gently, and the mix put in the dark for incubation for 15 min. In addition, 5 μL PI was added to the sample. The apoptotic cell rate was measured with a flow cytometer (Beckman Coulter, USA).

### Migration assay

Cell migration was evaluated by a modified two-chamber migration assay with a pore size of 8 μm. A cell suspension of 100 μL (around 2×10^5^ cells/mL) without serum was added to the upper transwell. Then, 600 μL culture medium with 10% FBS was added to the lower compartment of the 24-well transwell. A375 cells were maintained for 24 h at 37°C with humidified air containing 5% CO_2_. After incubation, cells at the upper surface of the filter were removed by a cotton swab, and the filter was fixed with methanol for 5 min. A375 cells at the lower surface of the filter were stained by Giemsa for 15 min. Cells were counted on a 100× microscope (Olympus CKX41, Japan).

### Cell transfection

To clarify the function of H19, pEX-H19 and its corresponding negative control (NC) pcDNA3.1 (GenePharma Co., China) were transfected into A375 cells. Pre-treated cells at the density of 2×10^5^ cells/well were seeded and incubated until the cells arrived at 70–80% confluence, and they were then transfected with pEX-H19 or NC by Lipofectamine 2000 reagent (Invitrogen, USA).

### Quantitative real time polymerase chain reaction (qRT-PCR)

Total RNA was obtained from A375 cells using Trizol reagent (Invitrogen). The One-Step SYBR^®^ PrimeScript^®^PLUS RT-RNA PCR kit (TaKaRa Biotechnology, China) was used for real-time PCR analysis to determine the expression level of H19. GAPDH was the internal control for H19.

### Western blot

Western blot was used in our study to detect protein expression. Protein was obtained from A375 cells using RIPA lysis buffer (Cat. No. R0010, Solarbio, China) supplemented with protease inhibitors (Thermo Fisher Scientific). The BCA™ protein assay kit (Pierce, USA) was used for determining proteins concentration. The western blot system was established by a Bio-Rad Bis-Tris Gel system following the manufacturer's instructions. Primary antibodies included: anti-cyclin D1 antibody (ab134175), anti-Bcl-2 antibody (ab32124), anti-Bax antibody (ab32503), anti-pro caspase 3 antibody (ab32150), anti-cleaved caspase-3 antibody (ab32042), anti-pro caspase-9 antibody (ab32539), anti-cleaved-caspase-9 antibody (ab2324), anti-matrix metalloproteinase (MMP)-9 antibody (ab73734), anti-MMP-2 antibody (ab37150), anti-phosphatidylinositol 3′-kinase (PI3K) antibody (ab191606), anti-phospho-PI3K antibody (ab182651), anti-protein kinase B (AKT) antibody (ab8805), anti-phospho-AKT antibody (ab8933), and anti-β-actin antibody (ab8227), all from Abcam (UK). Primary antibodies were prepared in 5% blocking buffer and diluted according to product instruction. These primary antibodies were incubated in membrane and maintained at 4°C overnight at the recommended concentration. For the second antibody incubation, cells were incubated with horseradish peroxidase (HRP) conjugated second antibody. Detection of signals and band intensity analyses were done by Image Lab™ Software (Bio-Rad, China).

### Statistical analysis

Data are reported as means± SD, based on at least three experiments. Statistical analyses were performed using Graphpad 6.0 statistical software (GraphPad, USA). P-values were calculated using a one-way analysis of variance (ANOVA) and Student's *t*-test. P values <0.05 were considered significant.

## Results

### SchA decreased cell proliferation and enhanced cell apoptosis in A375 cells

Firstly, an experiment was designed to determine the concentration at which SchA had the best effect in decreasing cell viability. As shown in Figure 2A, cells exposed to different concentrations of SchA (10, 20, 30, 40, and 50 μM) had significantly decreased viability with increasing concentrations of SchA compared with control (P<0.05, P<0.01 or P<0.001). SchA at the concentration of 30 μM was chosen for the subsequent experiments because 50.2% cell viability was close to EC_50_ under this concentration. BrdU assay was performed to detect cell proliferation and we found that SchA (30 μM) significantly decreased cell proliferation (P<0.01, Figure 2B). In addition, due to the close relationship between cyclin D1 and cell cycle, we found that SchA (30 μM) down-regulated cyclin D1 (P<0.05, Figure 2C) and enhanced cell apoptosis (P<0.001, Figure 2D). Moreover, we detected the accumulated level of apoptotic proteins, and found that cleaved-caspase-3 (P<0.001), cleaved-caspase-9 (P<0.001), and Bax (P<0.01) were up-regulated while Bcl-2 was down-regulated (P<0.05) by SchA (30 μM) compared with control (Figure 2E and F). Taken together, these findings indicate that SchA decreased cell proliferation and enhanced cell apoptosis.

**Figure 2.** A, Cell viability was detected under different schizandrin A (SchA) concentrations by Cell Counting Kit-8 assay. Cell proliferation (**B**) and (**C**) expression and level of cyclin D1 were analyzed via BrdU, western blot, and quantitatively, respectively. **D**, Cell apoptosis was analyzed by flow cytometry. Cell apoptosis-related proteins were detected by western blot (**E**) and quantitatively (**F**). β-actin was used as control. Data are reported as means±SD (n=3). *P<0.05, **P<0.01, and ***P<0.001 compared to control (ANOVA and Student's *t*-test).

### SchA decreased cell migration in A375 cells

In MM, migration is one of the main approaches for tumor metastasis (14). Hence, we detected the effect of SchA (30 μM) on cell migration. As shown in Figure 3A, SchA decreased cell migration (P<0.01) compared with control. In addition, it is well known that MMP-2 and MMP-9 are involved in cell migration (15), and therefore, we determined their accumulated levels. Interestingly, we found that MMP-9 and MMP-2 were significantly down-regulated by SchA compared with control (both P<0.05, Figure 3B and C). Thus, SchA showed ability in decreasing cell migration.

**Figure 3.** Schizandrin A (SchA) decreased cell migration. **A**, Cell migration was detected by transwell two-chamber assay. **B**, MMP-2 and MMP-9 protein levels were determined by western blot. **C**, Levels of MMP-2 and MMP-9 were analyzed quantitatively. β-actin was used as control. Data are reported as means±SD (n=3). *P<0.05 and **P<0.01 compared to control (Student's *t*-test).

### SchA negatively regulated the expression of H19

Previous research has reported that lncRNA H19 has shown tumor-promoting effects in multiple tumors (11). In our study, we explored whether H19 was dysregulated in A375 cells. Results showed that SchA (30 μM) significantly down-regulated the expression of H19 in A375 cells compared with control (P<0.01, Figure 4). This information hinted that H19 might participate in SchA's tumor-suppressive effects.

**Figure 4.** Schizandrin A (SchA) down-regulated H19 in A375 cells via qRT-PCR. Data are reported as means±SD (n=3). **P<0.01 (Student's *t*-test).

### SchA inhibited cell proliferation and increased cell apoptosis through down-regulation of H19

To identify the mechanism by which SchA regulated cell proliferation and apoptosis, pEX-H19 was transfected into A375 cells. The significant up-regulation of H19 after transfection with pEX-H19 indicated high transfection efficiency (P<0.01, Figure 5A). Then, we detected the effects of overexpression of H19 on cell proliferation and cell apoptosis. Results showed that transfection with pEX-H19 increased cell proliferation (P<0.01, Figure 5B), up-regulated cyclin D1 (P<0.05, Figure 5C), and decreased cell apoptosis (P<0.01, Figure 5D) compared with pEX group. In addition, the apoptotic proteins cleaved-caspase-3 (P<0.05), cleaved-caspase-9 (P<0.05), and Bax (P<0.05) were down-regulated while Bcl-2 was up-regulated (P<0.05) after transfection with pEX-H19 compared with the group transfected with pEX (Figure 5E and F). In summary, we inferred that SchA decreased cell proliferation and enhanced cell apoptosis via down-regulation of H19.

**Figure 5.** Schizandrin A (SchA) decreased cell proliferation and increased cell apoptosis via down-regulation of H19. **A**, Overexpression of H19 was established through transfection with pEX-H19 in A375 cells. Cell proliferation (**B**) and (**C**) expression and level of cyclin D1 were analyzed via BrdU, western blot, and quantitatively, respectively. **D,** Cell apoptosis was analyzed by flow cytometry. Cell apoptosis-related proteins were detected by western blot (**E**) and analyzed quantitatively (**F**). β-actin was used as control. All data are reported as means±SD (n=3). *P<0.05, **P<0.01 and ***P<0.001 compared to control or as indicated (ANOVA and Student's *t*-test).

### SchA decreased cell migration via down-regulation of H19

Similarly, we detected the effect of H19 overexpression on cell migration. We found that co-treatment with SchA and H19 overexpression increased cell migration (P<0.05, Figure 6A) as well as MMP-2 and MMP-9 expression (both P<0.05, Figure 6B and C) compared with co-treatment with SchA and transfection with pEX. Thus, we found that SchA decreased cell migration via down-regulation of H19.

**Figure 6.** Schizandrin A (SchA) decreased cell migration by down-regulating H19. **A**, Cell migration was detected by transwell two-chamber assay. MMP-2 and MMP-9 protein levels were detected by western blot (**B**) and analyzed quantitatively (**C**). β-actin was used as control. Data are reported as means±SD (n=3). *P<0.05 and **P<0.01 compared to control or as indicated (ANOVA and Student's *t*-test).

### SchA inactivated PI3K/AKT pathway by down-regulation of H19

PI3K/AKT was reported to be involved in MM (16). Hence, we investigated the effects of SchA on this pathway. Results demonstrated that SchA down-regulated the phosphorylation of PI3K (P<0.001) and AKT (P<0.05) while co-treatment with SchA and H19 overexpression led to the opposite results (P<0.01, Figure 7A and B). Thus, SchA might inhibit PI3K/AKT pathway through down-regulation of H19.

**Figure 7.** Schizandrin A (SchA) inhibited PI3K/AKT through down-regulation of H19. **A**, Phosphorylation of PI3K and AKT was detected by western blot. **B**, Levels of p/t-PI3K and p/t-AKT were analyzed quantitatively. β-actin was used as control. Data are reported as means±SD (n=3). *P<0.05, **P<0.01, and ***P<0.001 compared to control or as indicated (ANOVA).

## Discussion

MM is a catastrophic skin cancer with aggressive biological actions, resistance to chemotherapy, and poor results (2). MM has a complex progress and it is hard to fully elucidate the underlying mechanisms. Hence, we used A375 cells to construct an *in vitro* cell model and investigated the effects of SchA on A375 cells. Results demonstrated that SchA decreased cell proliferation and migration, increased cell apoptosis, and inhibited PI3K/AKT signaling pathway through down-regulating lncRNA H19.

Cell line A375 is often used for the *in vitro* model of MM (17). Firstly, we explored the effects of SchA on cell viability and cell proliferation. Results showed that SchA significantly decreased cell viability in a dose-dependent manner. Moreover, BrdU assay demonstrated that SchA significantly alleviated cell proliferation. Our study was consistent with the previous study that SchA inhibited cell proliferation in breast cancer cells (18). Furthermore, previous studies have reported that cyclin D1 is an important proto-oncogene that is upregulated in multiple cancers, such as breast, prostate, and MM (19,20). Cyclin D1 exerts important functions in regulating cell proliferation via activation of cyclin-dependent kinases (19). In our study, we found that SchA inhibited the accumulation of cyclin D1, which is consistent with the findings of Kim et al. (18) that SchA decreases cell proliferation by regulating cell cycle-related proteins, such as cyclin D1.

In addition, it is well-known that apoptosis plays important roles in cancer cells, and apoptosis related proteins are considered a promising target for molecule-based pharmacological intervention (21). SchA increased cell apoptosis in our study. Moreover, caspase-3, caspase-9, Bcl-2, and Bax are all apoptosis-related proteins (22). Our study revealed that SchA up-regulated the expression of pro-apoptotic proteins cleaved-caspase-3, cleaved-caspase-9, and Bax while it down-regulated the expression of anti-apoptotic protein Bcl-2. Our findings were consistent with the study of Kim et al. (23) that SchA extract induced apoptosis presented by the down-regulation of Bcl-2 and up-regulation of Bax, cleaved-caspase, and cleaved-caspase-9.

Furthermore, migration of cells to surrounding tissues is one of the initial and critical steps in the progression of cancer metastasis. Metastasis is the most important cause of cancer-related death (24). Therefore, we detected the effects of SchA on cell migration and found that it significantly decreased cell migration, suggesting it might have functions in inhibiting MM metastasis. Moreover, MMP-2 and MMP-9 are two important factors in cell migration and their overexpression is often related to poor progression in cancer (25). In our study, SchA decreased MMP-2 and MMP-9 expression, indicating the inhibition effects of SchA in the progress of MM.

Increasing evidence suggested that lncRNAs acted as molecular switches to regulate cell proliferation, cell apoptosis, and cell migration (26). Among the identified lncRNAs, H19 was observed to be essential for human tumor growth (27), including bladder cancer (27), colorectal cancer (28), gastric cancer (29), and MM (12). In our study, we found that SchA inhibited the expression of H19, suggesting that H19 might be involved in the inhibition effects of SchA on A375 cell growth and migration.

To alter the expression of H19, pEX-H19 was transfected into A375 cells. The results showed that co-treatment and transfection with pEX-H19 and SchA blockaded the effects of SchA on A375 cells as evidenced by increasing cell proliferation and migration, and inhibiting cell apoptosis. This is consistent with previous findings that H19 enhances breast cancer cell proliferation (30) and elevated H19 promotes bladder cancer proliferation (31). In addition, lncRNA H19 promotes cell migration in cholangiocarcinoma (32). Moreover, Zhu et al. (33) found that H19 knockdown increased the rate of apoptosis in ovarian cancer cells, which was the same trend as our study. Our study was the first to demonstrate that SchA played its roles in A375 cells through regulation of H19.

PI3K/AKT signaling pathway has been reported to play important roles in cell proliferation, survival, and metabolism (34), and was observed to be closely associated with MM (35). In our study, SchA decreased the phosphorylation level of PI3K and AKT, indicating that SchA inactivated PI3K/AKT signaling pathways. On the other hand, overexpression of H19 activated PI3K/AKT pathway. Previous studies proved that activation of PI3K/AKT was often related to the promotion of cancer progression while inactivation of PI3K/AKT was involved in inhibiting cancer development (36). These results demonstrated that SchA might inhibit A375 cell growth through inhibiting PI3K/AKT pathway.

### Conclusions

Our study demonstrated that SchA inhibited proliferation and migration of melanoma A375 cells, and increased apoptosis and inhibited PI3K/AKT pathway through down-regulation of lncRNA H19. Our study may lay the foundation for the study of MM in the future.
